This article has been retracted.

# Diaqua­bis(pyridine-2-carboxyl­ato-κ^2^ *N*,*O*)iron(II)

**DOI:** 10.1107/S1600536809005765

**Published:** 2009-02-25

**Authors:** Guohua Xia, Zexi Sun

**Affiliations:** a Institute of Applied Materials, College of Resource & Environmental Management, Jiangxi University of Finance & Economics, Nanchang, Jiangxi 330013, People’s Republic of China; b Department of Chemistry, College of Chemistry and Chemical Engineering, Xiamen University, Xiamen, Fujian 361005, People’s Republic of China

## Abstract

The Fe^II^ atom in the title complex, [Fe(C_6_H_4_NO_2_)_2_(H_2_O)_2_], exists in a distorted octa­hedral coordination geometry defined by two O and two N atoms from two pyridine-2-carboxyl­ate ligands and two O atoms of two water mol­ecules. In the crystal structure, mol­ecules are linked into a three-dimensional framework by O—H⋯O hydrogen bonds.

## Related literature

For the design and construction of metal-organic supramolecular structures, see: Desiraju (1997 ▶); Braga *et al.* (1998 ▶); Mccann *et al.* (1996 ▶); Wai *et al.* (1990 ▶); Yaghi *et al.* (1996 ▶); Min & Lee (2002 ▶); Maira *et al.* (2001 ▶). For bond-length data, see: Allen *et al.* (1987 ▶).

## Experimental

### 

#### Crystal data

[Fe(C_6_H_4_NO_2_)_2_(H_2_O)_2_]
*M* *_r_* = 336.09
Monoclinic,
*a* = 11.6255 (3) Å
*b* = 9.0247 (4) Å
*c* = 14.9724 (2) Å
β = 105.568 (2)°
*V* = 1513.22 (8) Å^3^
*Z* = 4
Mo *K*α radiation
μ = 1.02 mm^−1^
*T* = 293 K
0.23 × 0.19 × 0.07 mm

#### Data collection

Bruker SMART APEX area-detector diffractometer
Absorption correction: multi-scan (*SADABS*; Sheldrick, 1996 ▶) *T*_min_ = 0.796, *T*_max_ = 0.928
10191 measured reflections
3283 independent reflections
2158 reflections with *I* > 2σ(*I*)
*R*_int_ = 0.043

#### Refinement

*R*[*F* ^2^ > 2σ(*F* ^2^)] = 0.051
*wR*(*F* ^2^) = 0.166
*S* = 1.08
3283 reflections
201 parameters
6 restraints
H atoms treated by a mixture of independent and constrained refinement
Δρ_max_ = 0.72 e Å^−3^
Δρ_min_ = −0.47 e Å^−3^

### 

Data collection: *SMART*  (Siemens, 1996 ▶); cell refinement: *SAINT* (Siemens, 1996 ▶); data reduction: *SAINT*; program(s) used to solve structure: *SHELXS97* (Sheldrick, 2008 ▶); program(s) used to refine structure: *SHELXL97* (Sheldrick, 2008 ▶); molecular graphics: *SHELXTL* (Sheldrick, 2008 ▶); software used to prepare material for publication: *SHELXTL*.

## Supplementary Material

Crystal structure: contains datablocks I, global. DOI: 10.1107/S1600536809005765/at2725sup1.cif

Structure factors: contains datablocks I. DOI: 10.1107/S1600536809005765/at2725Isup2.hkl

Additional supplementary materials:  crystallographic information; 3D view; checkCIF report

## Figures and Tables

**Table:** 

Fe1—O1	2.163 (2)
Fe1—O2	2.148 (3)
Fe1—O3	2.164 (2)
Fe1—O5	2.154 (2)
Fe1—N1	2.262 (3)
Fe1—N2	2.279 (2)

**Table:** 

O1—Fe1—O2	84.52 (10)
O1—Fe1—O3	167.30 (9)
O1—Fe1—O5	98.68 (10)
O2—Fe1—O3	92.66 (10)
O2—Fe1—O5	95.00 (10)
O3—Fe1—O5	93.89 (9)
O1—Fe1—N1	86.39 (10)
O2—Fe1—N1	163.77 (12)
O3—Fe1—N1	99.03 (10)
O5—Fe1—N1	73.12 (9)
O1—Fe1—N2	93.92 (9)
O2—Fe1—N2	99.14 (10)
O3—Fe1—N2	74.26 (9)
O5—Fe1—N2	161.88 (9)
N1—Fe1—N2	94.86 (10)

**Table 2:** Hydrogen-bond geometry (Å, °)

*D*—H⋯*A*	*D*—H	H⋯*A*	*D*⋯*A*	*D*—H⋯*A*
O1—H1*B*⋯O4^i^	0.805 (18)	1.93 (2)	2.726 (3)	169 (4)
O1—H1*A*⋯O5^ii^	0.82	1.87	2.661 (3)	161
O2—H2*B*⋯O4^iii^	0.82 (5)	1.92 (5)	2.704 (3)	159 (6)
O2—H2*A*⋯O6^ii^	0.82	1.94	2.697 (4)	153

Symmetry codes: (i) ; (ii) ; (iii) .

## supplementary crystallographic information

### Comment

In the synthesis of crystal structures by design, the assembly of molecular units in predefined arrangements is a key goal (Desiraju, 1997; Braga *et al.*, 1998). Due to carboxyl groups are one of the most important classes of biological ligands, the coordination of metal-carboxyl groups complexes are of critical importance in biological systems, organic materials and coordination chemistry. Recently, carboxyl groups with variable coordination modes have been used to construct metal-organic supramolecular structures (Mccann *et al.*, 1996; Wai *et al.*, 1990; Yaghi *et al.*, 1996; Min & Lee 2002; Maira *et al.*, 2001). We report here in the crystal structure of the title compound, (I).

In the molecule of (I) (Fig. 1), the ligand bond lengths and angles are within normal ranges (Allen *et al.*, 1987). In the title complex, each Fe^II^ atom is axially coordinated by water molecules and consists of an equatorial plane of two oxygen donors and two nitrogen donors from two pyridine-2-carboxylato ligands with a distorted octahedral coordination geometry. The Fe—O bonds [average 2.152 (4) Å] are somewhat shorter than the Fe—N distances [average 2.270 (8) Å].

In the crystal structure, O—H···O hydrogen bonds (Fig. 2 and Table 2) seem to be effective in the stabilization of the structure, resulting in the formation of a supramolecular network structure.

### Experimental

Crystals of the title compound were synthesized using hydrothermal method in a 23 ml Teflon-lined Parr bomb, which was then sealed. Iron(II) chloride tetrahydrate (198.71 mg, 1 mmol), pyridine-2-carboxylic acid (246 mg, 2 mmol) and distilled water (10 g) were placed into the bomb and sealed. The bomb was then heated under autogenous pressure up to 433 K over the course of 7 d and allowed to cool at room temperature for 24 h. Upon opening the bomb, a clear colourless solution was decanted from small purple crystals. These crystals were washed with distilled water followed by ethanol, and allowed to air-dry at room temperature.

### Refinement

H1B and H2B (for two water molecules) were located in difference syntheses and refined isotropically [O—H = 0.805 (18) and 0.82 (5) Å, *U*_iso_(H) = 0.093 (15) and 0.18 (3) Å^2^]. The remaining H atoms were positioned geometrically, with O—H = 0.82 Å (for H_2_O) and C—H = 0.93 Å for aromatic H, and constrained to ride on their parent atoms, with *U*_iso_(H) = *xU*_eq_(C,*O*), where *x* = 1.2 for aromatic H atoms and *x* = 1.5 for all other H atoms.

### Crystal data

**Table:**

[Fe(C_6_H_4_NO_2_)_2_(H_2_O)_2_]	*F*(000) = 688
*M**_r_* = 336.09	*D*_x_ = 1.475 Mg m^−^^3^
Monoclinic, *P*2_1_/*n*	Mo *K*α radiation, λ = 0.71073 Å
Hall symbol: -P 2yn	Cell parameters from 2834 reflections
*a* = 11.6255 (3) Å	θ = 2.4–24.8°
*b* = 9.0247 (4) Å	µ = 1.02 mm^−^^1^
*c* = 14.9724 (2) Å	*T* = 293 K
β = 105.568 (2)°	Plane, purple
*V* = 1513.22 (8) Å^3^	0.23 × 0.19 × 0.07 mm
*Z* = 4	

### Data collection

**Table:**

Bruker SMART APEX area-detector diffractometer	3283 independent reflections
Radiation source: fine-focus sealed tube	2158 reflections with *I* > 2σ(*I*)
graphite	*R*_int_ = 0.043
φ and ω scans	θ_max_ = 27.3°, θ_min_ = 2.0°
Absorption correction: multi-scan (*SADABS*; Sheldrick, 1996)	*h* = −14→14
*T*_min_ = 0.796, *T*_max_ = 0.928	*k* = −11→11
10191 measured reflections	*l* = −19→18

### Refinement

**Table:**

Refinement on *F*^2^	Secondary atom site location: difference Fourier map
Least-squares matrix: full	Hydrogen site location: inferred from neighbouring sites
*R*[*F*^2^ > 2σ(*F*^2^)] = 0.051	H atoms treated by a mixture of independent and constrained refinement
*wR*(*F*^2^) = 0.166	*w* = 1/[σ^2^(*F*_o_^2^) + (0.089*P*)^2^ + 0.0485*P*] where *P* = (*F*_o_^2^ + 2*F*_c_^2^)/3
*S* = 1.08	(Δ/σ)_max_ = 0.001
3283 reflections	Δρ_max_ = 0.72 e Å^−^^3^
201 parameters	Δρ_min_ = −0.47 e Å^−^^3^
6 restraints	Extinction correction: *SHELXL97* (Sheldrick, 2008), Fc^*^=kFc[1+0.001xFc^2^λ^3^/sin(2θ)]^-1/4^
Primary atom site location: structure-invariant direct methods	Extinction coefficient: 0.0048 (16)

### Special details

**Table:**

Geometry. All e.s.d.'s (except the e.s.d. in the dihedral angle between two l.s. planes) are estimated using the full covariance matrix. The cell e.s.d.'s are taken into account individually in the estimation of e.s.d.'s in distances, angles and torsion angles; correlations between e.s.d.'s in cell parameters are only used when they are defined by crystal symmetry. An approximate (isotropic) treatment of cell e.s.d.'s is used for estimating e.s.d.'s involving l.s. planes.
Refinement. Refinement of *F*^2^ against ALL reflections. The weighted *R*-factor *wR* and goodness of fit *S* are based on *F*^2^, conventional *R*-factors *R* are based on *F*, with *F* set to zero for negative *F*^2^. The threshold expression of *F*^2^ > σ(*F*^2^) is used only for calculating *R*-factors(gt) *etc*. and is not relevant to the choice of reflections for refinement. *R*-factors based on *F*^2^ are statistically about twice as large as those based on *F*, and *R*- factors based on ALL data will be even larger.

### Fractional atomic coordinates and isotropic or equivalent isotropic displacement parameters (Å^2^)

**Table:**

	*x*	*y*	*z*	*U*_iso_*/*U*_eq_	
Fe1	0.74557 (4)	0.85895 (5)	0.62770 (3)	0.0492 (2)	
O1	0.8189 (2)	0.7456 (3)	0.75783 (16)	0.0565 (6)	
H1A	0.7646	0.7075	0.7752	0.085*	
O2	0.5913 (2)	0.8895 (3)	0.6788 (2)	0.0606 (7)	
H2A	0.5961	0.8351	0.7235	0.091*	
O3	0.65069 (19)	0.9271 (3)	0.48892 (15)	0.0527 (6)	
O4	0.5389 (2)	0.8582 (3)	0.35014 (17)	0.0592 (7)	
O5	0.8181 (2)	1.0762 (3)	0.66750 (16)	0.0540 (6)	
O6	0.9719 (3)	1.2298 (3)	0.6897 (2)	0.0772 (8)	
N1	0.9337 (3)	0.8594 (3)	0.6119 (2)	0.0534 (7)	
N2	0.6907 (2)	0.6454 (3)	0.54619 (18)	0.0435 (6)	
C1	0.6030 (3)	0.8306 (4)	0.4297 (2)	0.0454 (7)	
C2	0.6264 (3)	0.6693 (3)	0.4578 (2)	0.0418 (7)	
C3	0.5833 (3)	0.5536 (4)	0.3976 (2)	0.0561 (9)	
H3	0.5407	0.5724	0.3367	0.067*	
C4	0.6042 (3)	0.4112 (4)	0.4288 (3)	0.0587 (9)	
H4	0.5742	0.3320	0.3897	0.070*	
C5	0.6703 (3)	0.3863 (4)	0.5188 (3)	0.0580 (9)	
H5	0.6864	0.2900	0.5407	0.070*	
C6	0.7123 (3)	0.5052 (4)	0.5758 (2)	0.0530 (8)	
H6	0.7568	0.4880	0.6365	0.064*	
C7	0.9225 (3)	1.1079 (4)	0.6662 (2)	0.0538 (8)	
C8	0.9906 (3)	0.9877 (4)	0.6345 (2)	0.0514 (8)	
C9	1.1059 (3)	1.0068 (5)	0.6312 (3)	0.0731 (11)	
H9	1.1448	1.0967	0.6481	0.088*	
C10	1.1632 (4)	0.8908 (6)	0.6027 (4)	0.0974 (17)	
H10	1.2406	0.9023	0.5974	0.117*	
C11	1.1060 (4)	0.7585 (6)	0.5820 (4)	0.108 (2)	
H11	1.1452	0.6771	0.5659	0.130*	
C12	0.9911 (4)	0.7474 (5)	0.5854 (3)	0.0813 (13)	
H12	0.9510	0.6583	0.5686	0.098*	
H1B	0.8859 (15)	0.715 (5)	0.778 (3)	0.093 (15)*	
H2B	0.539 (5)	0.953 (5)	0.673 (4)	0.18 (3)*	

### Atomic displacement parameters (Å^2^)

**Table:**

	*U*^11^	*U*^22^	*U*^33^	*U*^12^	*U*^13^	*U*^23^
Fe1	0.0490 (3)	0.0448 (4)	0.0474 (3)	−0.0005 (2)	0.0020 (2)	−0.00062 (19)
O1	0.0430 (12)	0.0648 (16)	0.0542 (14)	0.0009 (12)	0.0002 (10)	0.0158 (11)
O2	0.0602 (15)	0.0518 (15)	0.0723 (18)	0.0102 (12)	0.0223 (13)	0.0148 (12)
O3	0.0536 (13)	0.0450 (14)	0.0507 (13)	−0.0018 (10)	−0.0013 (10)	0.0043 (10)
O4	0.0566 (14)	0.0563 (16)	0.0512 (14)	0.0076 (11)	−0.0091 (10)	0.0080 (10)
O5	0.0489 (13)	0.0466 (13)	0.0659 (15)	−0.0013 (10)	0.0144 (10)	−0.0088 (11)
O6	0.0798 (18)	0.0646 (18)	0.096 (2)	−0.0277 (15)	0.0388 (15)	−0.0312 (15)
N1	0.0535 (16)	0.0470 (18)	0.0624 (18)	−0.0004 (13)	0.0205 (13)	−0.0032 (13)
N2	0.0437 (13)	0.0411 (15)	0.0403 (14)	0.0004 (11)	0.0018 (10)	0.0027 (10)
C1	0.0345 (14)	0.054 (2)	0.0428 (17)	0.0025 (13)	0.0016 (12)	0.0015 (14)
C2	0.0361 (14)	0.0442 (18)	0.0418 (16)	−0.0003 (12)	0.0045 (11)	−0.0028 (13)
C3	0.0540 (19)	0.057 (2)	0.0473 (18)	0.0048 (16)	−0.0028 (14)	−0.0067 (16)
C4	0.059 (2)	0.047 (2)	0.065 (2)	0.0017 (17)	0.0074 (17)	−0.0142 (17)
C5	0.064 (2)	0.043 (2)	0.070 (2)	0.0023 (16)	0.0226 (18)	−0.0010 (16)
C6	0.0591 (18)	0.047 (2)	0.0489 (18)	0.0017 (16)	0.0080 (14)	0.0045 (15)
C7	0.059 (2)	0.057 (2)	0.0445 (18)	−0.0115 (16)	0.0121 (15)	−0.0065 (15)
C8	0.0509 (17)	0.058 (2)	0.0456 (17)	0.0039 (16)	0.0140 (13)	0.0021 (15)
C9	0.061 (2)	0.075 (3)	0.088 (3)	−0.008 (2)	0.029 (2)	−0.001 (2)
C10	0.070 (3)	0.095 (4)	0.143 (5)	0.002 (3)	0.055 (3)	0.007 (3)
C11	0.090 (3)	0.077 (3)	0.183 (6)	0.013 (3)	0.081 (4)	−0.007 (3)
C12	0.076 (3)	0.056 (3)	0.124 (4)	0.003 (2)	0.047 (3)	−0.007 (2)

### Geometric parameters (Å, °)

**Table:**

Fe1—O1	2.163 (2)	C1—C2	1.520 (4)
Fe1—O2	2.148 (3)	C2—C3	1.382 (4)
Fe1—O3	2.164 (2)	C3—C4	1.366 (5)
Fe1—O5	2.154 (2)	C3—H3	0.9300
Fe1—N1	2.262 (3)	C4—C5	1.379 (5)
Fe1—N2	2.279 (2)	C4—H4	0.9300
O1—H1A	0.8200	C5—C6	1.377 (5)
O1—H1B	0.805 (18)	C5—H5	0.9300
O2—H2A	0.8200	C6—H6	0.9300
O2—H2B	0.82 (5)	C7—C8	1.494 (5)
O3—C1	1.260 (4)	C8—C9	1.365 (5)
O4—C1	1.249 (4)	C9—C10	1.369 (6)
O5—C7	1.251 (4)	C9—H9	0.9300
O6—C7	1.247 (4)	C10—C11	1.361 (7)
N1—C12	1.329 (5)	C10—H10	0.9300
N1—C8	1.332 (4)	C11—C12	1.353 (6)
N2—C6	1.342 (4)	C11—H11	0.9300
N2—C2	1.351 (4)	C12—H12	0.9300
			
O1—Fe1—O2	84.52 (10)	N2—C2—C1	115.8 (3)
O1—Fe1—O3	167.30 (9)	C3—C2—C1	122.4 (3)
O1—Fe1—O5	98.68 (10)	C4—C3—C2	119.2 (3)
O2—Fe1—O3	92.66 (10)	C4—C3—H3	120.4
O2—Fe1—O5	95.00 (10)	C2—C3—H3	120.4
O3—Fe1—O5	93.89 (9)	C3—C4—C5	119.2 (3)
O1—Fe1—N1	86.39 (10)	C3—C4—H4	120.4
O2—Fe1—N1	163.77 (12)	C5—C4—H4	120.4
O3—Fe1—N1	99.03 (10)	C6—C5—C4	119.4 (3)
O5—Fe1—N1	73.12 (9)	C6—C5—H5	120.3
O1—Fe1—N2	93.92 (9)	C4—C5—H5	120.3
O2—Fe1—N2	99.14 (10)	N2—C6—C5	121.7 (3)
O3—Fe1—N2	74.26 (9)	N2—C6—H6	119.1
O5—Fe1—N2	161.88 (9)	C5—C6—H6	119.1
N1—Fe1—N2	94.86 (10)	O6—C7—O5	124.9 (3)
Fe1—O1—H1A	109.5	O6—C7—C8	119.1 (3)
Fe1—O1—H1B	128 (3)	O5—C7—C8	116.0 (3)
H1A—O1—H1B	119.0	N1—C8—C9	121.7 (3)
Fe1—O2—H2A	109.5	N1—C8—C7	116.3 (3)
Fe1—O2—H2B	136 (3)	C9—C8—C7	122.0 (3)
H2A—O2—H2B	112.5	C8—C9—C10	118.6 (4)
C1—O3—Fe1	119.6 (2)	C8—C9—H9	120.7
C7—O5—Fe1	120.9 (2)	C10—C9—H9	120.7
C12—N1—C8	118.8 (3)	C11—C10—C9	119.5 (4)
C12—N1—Fe1	127.4 (3)	C11—C10—H10	120.2
C8—N1—Fe1	113.8 (2)	C9—C10—H10	120.2
C6—N2—C2	118.7 (3)	C12—C11—C10	118.9 (4)
C6—N2—Fe1	128.3 (2)	C12—C11—H11	120.5
C2—N2—Fe1	113.04 (19)	C10—C11—H11	120.5
O4—C1—O3	124.8 (3)	N1—C12—C11	122.3 (4)
O4—C1—C2	118.1 (3)	N1—C12—H12	118.8
O3—C1—C2	117.0 (3)	C11—C12—H12	118.8
N2—C2—C3	121.8 (3)		

### Hydrogen-bond geometry (Å, °)

**Table:**

*D*—H···*A*	*D*—H	H···*A*	*D*···*A*	*D*—H···*A*
O1—H1B···O4^i^	0.81 (2)	1.93 (2)	2.726 (3)	169 (4)
O1—H1A···O5^ii^	0.82	1.87	2.661 (3)	161
O2—H2B···O4^iii^	0.82 (5)	1.92 (5)	2.704 (3)	159 (6)
O2—H2A···O6^ii^	0.82	1.94	2.697 (4)	153

Symmetry codes: (i) *x*+1/2, −*y*+3/2, *z*+1/2; (ii) −*x*+3/2, *y*−1/2, −*z*+3/2; (iii) −*x*+1, −*y*+2, −*z*+1.
